RETRACTED

# Individualized Assessment and Therapeutic Intervention for Mental Health of American Postmodern Novelists

**DOI:** 10.1155/2022/1277121

**Published:** 2022-06-29

**Authors:** Ningxia Qu

**Affiliations:** Anqing Normal University, School of Foreign Languages, Anhui, Anqing 246133, China

## Abstract

**Objective:**

Therapeutic intervention can improve the overall level of mental health of American postmodern fiction writers by improving their social communication skills and overall well-being. This paper discusses the application of art therapy in the mental health education of American postmodern novel creators and proves that expressive art therapy intervention is effective in improving the mental health level of American postmodern novel creators.

**Method:**

This article attempts to help American postmodernist novel creators understand their own mental health status by means of individualized assessment and therapeutic intervention and to analyze and discover their own potential mental health problems. The writers of postmodernist novels in the USA were measured and screened by means of scales and questionnaires, and the members who met the experimental intervention were divided into experimental group and control group, and the experimental group received a 30-day reception music therapy intervention. After the intervention, the data will be counted, and the quantitative and qualitative aspects will be analyzed to comprehensively evaluate the effect of the intervention. *Results/Discussion*. Receptive music therapy intervention has a significant effect in relieving the anxiety of American postmodernist novel creators and plays a positive role in helping American postmodernist novel creators better adapt to study life and build good emotional psychology and interpersonal relationships. Psychological counseling relies more on external forces to correct cognition and adjust psychology, while music therapy intervention, as a nonsemantic art, can arouse inner functions and mobilize the self-healing potential of American postmodern novel creators. Practice has proven that when the language intervention of traditional psychotherapy encounters resistance and silence, music as a special language plays a vital role. The nonlinguistic nature of music, through a mode of reproduction of sounds in nature, makes the beautiful and soothing melody stimulate a pleasant and peaceful psychological experience through human hearing.

## 1. Introduction

The American postmodernist trend of thought, with its emphasis on the retreat of grand narratives and the dissolution of deep models, the deconstruction of microscopic subjects, the migration from diachronic to synchronic, and the aestheticization of daily life, has completely broken through the more integrated mainstream discourse in the past [1]. Boundaries, such as dispelling the center, questioning rationality, and advocating the humanities care of diversified value tendencies, with the attitude of “subversion,” “criticism,” and “dissolution,” not only strongly impact people's knowledge and understanding of the world, but also profoundly affect the perspective of grasping and expressing the world in literary and artistic creation [2].

RETRACTED

The introduction of American postmodernism, especially its literary and cultural trends, has provided a new idea and a broad vision for the development of literature in the new era [3]. It comprehensively promotes the renewal and transformation of literary concepts in the new era, liberates contemporary literary creators and researchers from the shackles of the original one-dimensional political ideology, and provides them with new personalization and diversification. To a certain extent, it has contributed to the development of diversification and complexity of literary creation and research in the new era and has a profound understanding of the philosophical spirit and the philosophical spirit of contemporary literature. The rise in stylistic awareness has had a unique impact.

Expressive art therapy uses the form of art to balance people's inner world and outer world through the process of art appreciation, art creation, art expression, and other psychological interventions to achieve unity [4]. At present, the use of music therapy intervention and painting therapy in expressive art therapy also gradually involves the mental health problems of American postmodern novel creators [5].

Medical institutions have successively set up music therapy intervention rooms and have begun enthusiastic exploration of music therapy interventions [6]. The Music Therapy Intervention Society, which regularly holds national music therapy intervention academic conferences, was established, which has contributed to the exchange and development of music therapy intervention scholars [7]. Taiwanese music therapy interventionist returned from the USA for the first time as a music therapy interventionist at the Taipei Xinai American Postmodernist Novel Creator Development Center and brought systematic and scientific music therapy intervention to Taiwan for the first time [8]. Afterwards, dozens of music therapy intervention masters who studied abroad returned to Taiwan to work. Most of them were registered music therapy interventionists in developed countries or regions including the USA [9]. Taiwan established the “Applied Music Promotion Association,” and with these returnees as the backbone, various lectures and classes were held, which made great achievements in promoting the cause of music therapy intervention in Taiwan. Compared with the mainland, Taiwan has entered the field a little later and has a different way of development. The scale of music therapy intervention is small, but it is small and sophisticated, relatively more professional, and has developed rapidly [10–12]. This paper presents the concept of applying visual analytics techniques to mental health assessments. According to the analysis results of different American postmodernist novel creators, suggestions for improvement can be given for different evaluation results.

RETRACTED

Music therapy intervention itself is the art of communication. Through continuous and effective improvement of therapeutic techniques, the therapist establishes a therapeutic relationship with the patient, which can improve the therapist's interpersonal skills. In the process of participating in music therapy intervention, American postmodern novel creators adjust unreasonable anxiety, change cognition, release pressure, and relieve mood, so as to adjust and improve tension and anxiety.

## 2. Methods

### 2.1. Mental Health Assessment Scale

The scales can be divided into numerical rating scales, standard rating scales, check-and-choice scales, and forced-choice rating scales according to the way the scale items are compiled. According to the nature of the rater, it can be divided into self-assessment and other assessment. According to the content of the scale, it can be divided into some clinical manifestations of neurology, social and interpersonal relationships, mental health, and behavioral problems. Here is a brief description of the mental health assessment scale according to the single symptom assessment scale and the comprehensive mental health assessment scale.

The single symptom assessment scale is designed to evaluate and analyze a specific psychological symptom of the subject. Compared with the single symptom assessment scale, the comprehensive mental health scale is more widely used in clinical practice. The comprehensive mental health scale helps individuals understand their own mental health from multiple aspects and maximizes their relevance to people's reality. In real life, common comprehensive mental health scales include SCL-90 symptom self-rating scale, Minnesota multiphasic personality test series, and psychosomatic health scale.

### 2.2. SCL-90 Symptom Self-Rating Scale

The SCL-90 symptom self-rating scale is suitable for adults over 16 years old. It can help individuals understand their own mental health from the aspects of emotion, thinking, consciousness, and living habits. People on the fringe have good discrimination, but not for people with mania and schizophrenia. The 10 factors and their reflections are shown in Table 1.

RETRACTED

### 2.3. Data Processing Method

The purpose of data processing is to filter and derive valuable and meaningful data from a large amount of disorganized data. In this paper, the SCL-90 symptom self-rating scale data is collected, stored, retrieved, processed, transformed, and transmitted as basic data.

#### 2.3.1. Data Organization

Data organization refers to the process of merging, storing, and processing data according to certain methods and rules and is often used in the establishment of systems. JSON (JavaScript object notation), CSV (comma-separated values), and XML (extensible markup language) are three data transmission formats commonly used in web systems.

JSON is based on a subset of ECMAScript and is a lightweight data interchange format. JSON has the advantages of concise, clear hierarchical structure, easy to read and write, easy to parse and generate, and improve network transmission efficiency, and JSON can represent any type of data.

The advantages and convenience of JSON make it an ideal data exchange language and a commonly used web data transmission format.

A CSV file consists of any records, separated by newlines, each record consists of attributes, and commas or tabs are often used as attribute separators to separate each attribute. CSV has the advantages of easily transferring table data between programs and having a smaller data volume when transferring the same amount of data and is suitable for storing cubes.

The system in this paper is a web system, using the SCL-90 symptom self-rating scale data as the basic data for collection and using the mySQL database to store the data. In order to facilitate the storage and reading of data, this article uses JSON as the data transmission format.

#### 2.3.2. Data Cleaning

Data cleaning is a very important step in data preprocessing. It removes the “dirty” data from the data and leaves valuable data. Before storing the SCL-90 scale data, this paper firstly evaluates the quality of the data, then cleans the data, and finally stores the valuable data in the database. Data cleaning refers to finding and correcting invalid values and vacancies in data, including many complex operations such as data standardization and normalization.

#### 2.3.3. Data Structure

A data structure is a collection of data elements that have one or more specific relationships to each other. In order to better evaluate the mental health of individuals, this paper needs to store the data of each evaluation of American postmodern novel creators, so as to comprehensively analyze the mental health of American postmodern novel creators in a certain period of time.

RETRACTED

The database of this paper contains three tables, namely: the information table of American postmodernist novel creators (userInfo), the basic data table (dataStore), and the result table (result). American postmodernist novel creator information table (userInfo) contains basic information such as gender, age, province, and occupation of American postmodernist novel creators, and the basic data table (data Store) contains the SCL-90 symptom self-rating scale. The results table (result) stores the evaluation results of American postmodern novel creators and the results after feature selection algorithm analysis.

### 2.4. Feature Selection Method

This paper introduces the existing feature selection algorithms from two aspects: whether the feature is divergent or not and the correlation between the feature and the target and explains the applicable situations of each algorithm. Among them, when choosing the logistic regression model based on L1 regularization or L2 regularization to select the features of this paper, the similarities and differences of the two regularized logistic regression models in the model training process are analyzed. In the training process of the model, the value of the feature coefficient *w* is different, resulting in different final weight feature vectors. L1 regularization only retains some features that are more relevant to the target at the end. Finally, the next set of more scattered features is preserved. In practical applications, the selection is made according to the specific needs analysis. If you only want to retain the features with greater influence, you can choose L1 regularization; and if only some features are not specially required to be retained, then L2 regularization can usually be obtained.

The variance selection method selects features according to the divergence of each feature and target. When analyzing the historical data of American postmodern novel creators, the variance selection method can be used to select American postmodern novel creators who fluctuate more. Factors and problems, that is, the factors and problems that American postmodernist novel creators are most susceptible to, then determine the threshold rule based on repeated experiments and finally determine the threshold using the mean variance as the variance selection method.

The logistic regression model of L1 regularization can retain the features with greater influence, and the logistic regression model based on L1 regularization is used to screen out the factors and problems that are highly correlated with the target; that is, the creators of American postmodern novels are always in the sub-mode. When there is more historical data on American postmodern novel creators, the results obtained by analyzing the data using a logistic regression model based on L1 regularization are more consistent with reality.

RETRACTED

When the historical data of American postmodernist novel creators is small, the results of the selection of factors and questions by the variance selection method are not accurate enough, and more features than the actual results are often obtained. The selected features are less than the actual results. By using the data of different American postmodernist novel creators to conduct experiments, and analyzing and learning the experimental results, it is finally found that when the number of historical data records of American postmodernist novel creators is less, the results selected by the regression model are prone to fluctuations, and the accuracy of the results is low. Combining the data analysis results of the creators of American postmodernist novels and the assessment time of the scale, the final determination is based on the time of one month; that is, when the number of historical data records of the creators of American postmodernist novels is greater than 5 times, the variance is used. A selection method and an L1-regularized-based logistic regression model were used to analyze historical data on American postmodern fiction writers.

The mental health assessment system in this paper combines the fluctuation characteristics selected by the variance selection method and the main characteristics selected by the logistic regression model based on L1 regularization as the characteristics that the creators of American postmodernist novels need to pay attention to. When the recorded data of the creators of American postmodernist novels is less than 5 times, the system counts the number of times the factors and problems fall into an unhealthy state each time and selects the features whose occurrence times are greater than the average number of records as the creation of American postmodernist novels.

## 3. Results

### 3.1. Analysis of Influencing Factors of Mental Health

#### 3.1.1. Correlation Analysis between Demographic Data and SCL-90 Factors

In order to understand the relationship between the demographic data and the mental health of the control group and the experimental group, we conducted a Pearson correlation analysis between the SCL-90 factors of the demographic data. The results of the control group analysis are shown in Figure 1. The psychological analysis results of the experimental group are shown in Figure 2.

RETRACTED

#### 3.1.2. Correlation Analysis between the Coping Style of the Control Group and the Experimental Group and Various Factors of SCL-90

Figures 3 and 4 show that there is a big difference in the SCL-90 factor scores and positive coping styles of the control group and the experimental group members.

### 3.2. Quantitative Analysis of Intervention Results

Two sets of questionnaires were used to conduct data statistics on the experimental group and the control group again, and the results of the two groups after the experiment were as follows.

Table 2 shows that after the intervention, the scores of the SAS anxiety self-rating scale in the experimental group decreased significantly, and the posttest scores were lower than the pretest scores, with significant differences. There was also a decrease in the scores of the control group, but there was no significant difference between the posttest scores and the pretest scores.

Table 3 shows that after the intervention, the scores of the self-rating depression scale in the experimental group decreased significantly, and the posttest scores were lower than the pretest scores, with a significant difference. The scores of the control group also decreased, but the scores were not as significant as those of the experimental group, and there was a significant difference.

Figure 5 shows that there is a significant difference in the scores of the experimental group and the control group. The scores of the experimental group were lower than those of the control group on the depression scale.

### 3.3. Qualitative Analysis of Intervention Results

Qualitative research is a research method in which the subject and the subjects discuss and communicate with each other. The goal of the research is to explore the impact of the behavior from the psychology and behavior of the subjects.

In this study, the author used a questionnaire in the form of a return visit to summarize and study the actual effect after the intervention by communicating with 50 American postmodernist novel creators in the intervention group and combining audio-visual materials. In the intervention activity, the participants reported their different feelings and gains in the questionnaire. Through the return visit, the overall activity went well without any harm or negative emotional impact on the creators of American postmodernist novels. The overall evaluation was good, and the evaluation feedback data is described below. The feedback evaluation scores of the intervention group after treatment are shown in Figure 6.

The overall satisfaction of the intervention group with the music therapy intervention was high, and they affirmed the form of music therapy intervention to relieve tension and anxiety. Writers of American postmodernist novels not only learned to adjust their anxiety during activities, but also learned how to get along with people during group intervention, narrowing the distance between people and improving their interpersonal skills.

RETRACTED

### 3.4. Overall Analysis of Intervention Outcomes

After 30 days of treatment intervention, the analysis of the anxiety data of the experimental group showed that there was a significant difference in the *T* value between the pretest and the posttest, the posttest score was significantly lower than the pretest score, and the anxiety value fell back to the normal mean. The music therapy intervention has a significant effect on relieving adjustment anxiety. The pretest and posttest scores of the control group did not decrease significantly, and there was no significant difference. Although they decreased, they were still at the critical value of mild anxiety. After analyzing the depression data of the experimental group, it was found that the values of the pretest and the posttest constituted a significant difference.

The intervention effect of female creators is more significant than that of male creators, which is related to women's strong suggestibility, and female creators are more easily affected by the intervention of music therapy intervention. Through the communication and feedback of American postmodernist novel creators after treatment, female creators are more likely than male creators to produce effects in their musical imagination and cause resonance.

Female creators adapt more obviously than male creators, and their scores tend to be more stable. It can be seen that female creators are more easily affected by emotional rendering and more likely to resonate emotionally than men, and the intervention effect is more obvious.

In addition, whether the recitation of the introductory language has a soft melody and cadence, as well as a friendly tone or the subject's charisma, all have an impact on the intervention effect.

#### 3.4.1. Promote Physical and Mental Relaxation and Awaken Inner Emotions

Through the peak experience, most of the creators' tense body and mind have been relaxed, and the pressure has been relieved. Some creators said they thought a lot of comfortable things and were relieved from the complicated real life. Through the catharsis of music, the creator calmed down and communicated with his heart in the process. The overall feeling was good, and he could learn to release pressure through relaxation.

In the feedback questionnaire before the treatment, the author learned that the anxiety value caused by sleep disorders is relatively high, and the dormitory work and rest time and individual sleep habits are different, which are easy to make American postmodernist novel creators produce anxiety. In addition, intensive study and busy green also have little time to communicate and talk with their own hearts, and it is easy to form resistance and pressure over time.

RETRACTED

Although music cannot change the reality, it can inject energy into the subjects, stimulate people's self-healing potential, and enhance people's confidence. By listening to music, they can enter the station of the soul, so that the soul can rest and the positive potential of the heart can be repaired.

#### 3.4.2. Vent Negative Emotions and Change Bad Cognitions

The writers of American postmodern novels are relatively fragile in emotional management and regulation, and the problems are more prominent. After the intervention of musical imagination, the creators of American postmodernist novels released the pressure in their hearts. The music mobilized the thoughts and passions of the creators of American postmodernist novels. The deep music brought inner peace, and the sound of the waves of the sea, specifically the rushing sound of the waves, washes away the inner thoughts, and the sea swallows up the unhappy emotions and guides the American postmodernist novel creators to imagine happier things. It is precisely the synesthesia effect with the previous experience that the music stimulates the synesthesia deep in the heart and plays the role of catharsis.

#### 3.4.3. Improve Communication Skills and Rebuild Self-Confidence

The creators of American postmodernist novels realized that interpersonal communication is an indispensable part, but in the process, due to the characteristics of doubt, avoidance, and distrust of the object of conversation, they also showed a self-closed side in their hearts. They are eager to pour out their inner world to others, but lack the social skills to communicate with others.

The rhythmic game and warm-up training, as well as the exchange and sharing discussion sessions, have promoted the opportunity to communicate with other members and enhanced everyone's understanding. The form of sharing and discussion-style music therapy intervention strengthens the communication between people, increases the sense of identity and closeness among team members, and understands that when dealing with people, we should learn to empathize and treat others leniently.

## 4. Discussion

### 4.1. Discussion on the Reliability and Validity Test of the Scale

#### 4.1.1. Item Screening of the Scale

Some scholars pointed out that the selection of items needs to comply with the principles of good certainty, good representativeness, strong independence, high sensitivity, and great importance [13–15]. The preparation of this questionnaire is divided into two steps. First, ask experts and psychology teachers to analyze the first edition of the American Postmodern Novel Creators Mental Health Questionnaire item by item, delete or revise the items that are difficult to understand, weak in representation, unclear in meaning, and repeated, so as to preliminarily ensure the validity of the items. The second step is to determine the form of the questionnaire from the aspects of the research scope, objects, and analysis methods [10, 16].

6 American postmodernist novel creators with good language ability and hearing impairment were asked to answer the entry, and the entry was modified according to the language habits of American postmodernist novel creators to fit the expression habits of American postmodernist novel creators. The certainty of the entry is guaranteed. Secondly, the correlation coefficient method was used to filter the items with the correlation coefficient between the item and the subscale total score greater than 0.3 as the cutoff value. The consistency between the item and the total score is greater than 0.3, indicating that the item has a good consistency with the total score and is representative of the relevant psychology. At the same time, it also shows that this item can evaluate the severity of the psychological problems of the subjects and has a high sensitivity. The correlation between items is significant, indicating that the items are independent.

RETRACTED

#### 4.1.2. Reliability

Test-retest reliability is used to examine the stability of the questionnaire across time. The specific method is that the same questionnaire is administered to the same subjects twice at different times. If the results of the two tests are consistent, the test-retest reliability of the questionnaire is good. General scale test-retest reliability correlation coefficient >0.7 indicates that the scale is stable and reliable [9, 17, 18]. The questionnaire was retested at two-week intervals, and the correlation coefficient of each subscale score ranged from 0.83 to 0.87. It shows that the test-retest reliability of the questionnaire is good [19, 20].

Reliability refers to the consistency, stability, and reliability of the questionnaire results. In this study, internal consistency reliability and test-retest reliability were used to investigate the questionnaire.

The questionnaire in this study includes five subscales, and there are uncorrelated contents among the subscales, so the internal consistency reliability of each subscale is calculated separately.

RETRACTED

Internal consistency reliability is often measured by Cronbach's *α* coefficient. Some scholars believe that *α* >0.8 indicates excellent internal consistency, *α* between 0.6 and 0.8 indicates better, and *α* <0.6 indicates poor [19].

#### 4.1.3. Validity

In this study, the school standard validity was used to examine the questionnaire. Calibration validity uses a recognized effective scale as the calibration standard to examine the correlation between the new scale and the results of the calibration scale [21, 22]. The larger the correlation coefficient, the better the validity of the new scale. In this study, SCL-90 was used as the calibration standard to examine the calibration-related validity of each subscale. The SCL-90 is a widely used mental health rating scale in the survey of the mental health of postmodern novel creators in the USA [23]. In this study, the depression subscale, anxiety subscale, obsessive-compulsive subscale, interpersonal sensitivity subscale, and hostile subscale were used as calibration standard, respectively, with the corresponding subscale of SCL-90. The correlation coefficients between the scores of the subscales of the American Postmodern Novel Creators Mental Health Questionnaire and the corresponding subscale scores of the SCL-90 ranged from 0.53 to 0.69, indicating that each subscale had good calibration validity.

### 4.2. The Role of Therapeutic Interventions on American Postmodern Fiction Writers

In traditional medical treatment and psychotherapy, American postmodernist novel creators cannot express all their emotions relaxedly and are subject to a lot of control [11, 24, 25]. Due to language limitations, it is difficult to express their emotions. In the intervention of art therapy, American postmodernist novel creators can fully express their hearts in pictures and works, and can express their emotions through proportion, layout, line, color, and content, which is impossible for other therapies [26–28]. It can make up for the blank of traditional therapy in inner emotional communication and has influence on the creators of American postmodernist novels.

#### 4.2.1. The Intervention of Art Therapy Can Build a Sense of Security for the Creators of American Postmodern Novels

In the process of art appreciation and expression, the main communication is through vision, without too much positional movement and language expression [22, 29, 30]. It is a relatively safe environment for American postmodern fiction writers with some communication barriers.

In terms of the expression of the paintings before and after, the artistic practice works of the creators of autistic American postmodernist novels have obviously changed in layout, from the layout of serious deviation at the beginning to the stable state of central layout later. In terms of the proportions of the picture, there is no serious imbalance, and the further to the back, the more stable and coordinated. These are all manifestations of the establishment of American postmodernist novel creators' sense of security [31].

RETRACTED

Although the creators of American postmodernist novels are different in the expression of pictures and changes in personal behavior, they have one thing in common; that is, they can stay in the classroom for a longer time and express in the form of painting and graffiti. They are more patient to express the picture completely. This relative calm is the expression of their sense of security, and the artistic expression is more detailed and complete.

#### 4.2.2. The Intervention of Art Therapy Contributes to the Emotional Expression of American Postmodernist Novelists

Compared with other courses, American postmodernist novel creators are more able to calm down in their artistic practice [32]. Regardless of whether they have been exposed to painting and handicraft, they all try to contact this material with less or less resistance.

In the embodiment of the works of American postmodernist novel creators, there can be a certain projection of life emotions, and they can express profoundly in their works [33]. Although American postmodernist novelists at this age cannot fully express their images, they can express their emotions more smoothly through shapes, colors, practice sequences, and movement characteristics in their artistic practice works [34].

After the negative emotions are vented many times, the creator's emotions will become relatively relaxed and stabilized. It was also reflected in the responses to the emotional questions of the questionnaire. Most American postmodernist novelists showed happy or calm emotions after art therapy intervention, and only a few did not show any special expressions.

The lower layout and repeated gravity graffiti are all manifestations of emotional repression and poor emotional management. This is very likely that the artistic experience of painting and other artistic experiences give the creators of American postmodernist novels the catharsis and management of emotions, so that they can let negative emotions such as anger and depression gradually ease, and they reduce aggressive and out-of-control behaviors.

#### 4.2.3. Art Therapy Can Improve the Self-Awareness and Observation Initiative of American Postmodern Novel Creators

Visual impact is extremely attractive to American postmodernist novelists. It is a special perception. Unlike vague and elusive verbal expressions, visual expressions are straightforward and simple, yet rich and clear. Therefore, the creators of American postmodern novels have a variety of visual perceptions when they study, which is very beneficial to their self-cognition ability [35]. The direct experience of images is much more effective than repeated repetition of words. At the same time, each time they appreciate and create a different visual form, this encourages them to continue to observe and obtain visual satisfaction [36].

RETRACTED

#### 4.2.4. Art Therapy Can Enhance the Emotional Communication between American Postmodern Fiction Writers and Others

When relatives and friends need to communicate with them, it is often because they do not care about the outside world and cannot use language smoothly for a while, which leads to difficulties in communicating with the outside world [37]. However, as art therapy interventions continue to advance, researchers can communicate with them more or less, and as the number of experiences increases, the communication becomes relatively frequent [38].

The weak perception of emotion by American postmodern novel creators makes it difficult for them to quickly get acquainted with anyone [23, 39]. They are unwilling to express their own world, and even less willing to enter the world of others. However, artistic expression becomes a medium of communication. In artistic practice, they express their inner feelings on the screen unconsciously [17, 25]. When their emotions are relatively stable, the therapist can discuss the content of the expression with him. At the same time, in their perception of more materials, they can gradually listen to the therapist's praise and begin to have certain eye contact. It is reflected from the questionnaire that five more American postmodernist novel creators began to express the content of their works. Two of them expressed their works in language, and three of them expressed more eyes and expressions and less verbal expressions. There are also 2 American postmodern novelists who have not started communicating, but the data is very reassuring. For example, in the later practice, after the parents came in, several children could say a few words to explain their works, instead of putting them aside and doing nothing.

## 5. Conclusion

Music therapy intervention exerts its nonsemantic function, which makes it difficult to express the way of expressing the entangled mentality that cannot be described in words. Therefore, the music therapy intervention method has incomparable advantages compared with other psychological counseling methods that rely solely on language, and the music therapy intervention has the characteristics of safety, greenness, and no side effects. Therefore, compared with traditional psychological counseling, music therapy intervention has a unique effect on solving communication disorders. Music therapy intervention is to use the nonverbal characteristics shared by music and the subconscious mind, with the help of music meditation and consciousness transformation, to deeply portray a positive inner image of the mind, to promote the release of subconscious activities, to correct psychological problems, and to stimulate self-healing potential. Music is the language of the subconscious mind. The language of the subconscious mind is much broader than the realm of consciousness. You can forget yourself in the language of the subconscious mind, and release yourself in the vast subconscious space through the function of musical imagination. You can listen to the music with your heart and be immersed in the situation, which will lead to an introspective peak experience, and then help the creators of American postmodern novels to achieve self-improvement.

RETRACTED

## Figures and Tables

**Figure 1:** Pearson correlation analysis results of mental health and demographic data in the control group.

**Figure 2:** Pearson correlation analysis results of mental health and demographic data in the experimental group.

**Figure 3:** The weights of each factor of SCL-90 in the coping style of the control group.

**Figure 4:** Coping style of the experimental group and the weight of each factor of SCL-90.

**Figure 5:** Comparison of scale scores between the experimental group and the control group.

**Figure 6:** Feedback evaluation scores after treatment in the intervention group.

**Table 1:** Interpretation of each factor of SCL-90 symptom self-rating scale.

Factor items	Reflect symptoms
Obsessive-compulsive symptoms	It mainly reflects the compulsive psychology of the subjects in life
Depression	It mainly reflects the subjects' depressed emotions and moods
Paranoid	It mainly reflects the subjects' delusions, suspicions
Hostility	It mainly reflects the hostile emotions of the subjects
Psychotic	It mainly reflects whether the subjects have various acute symptoms and behaviors, mainly including the detection of schizophrenia items
Fear	It mainly reflects the fear of the subjects about traveling
Somatization	Mainly reflects the subject's physical discomfort
Anxiety	It mainly reflects the irritability
Interpersonal sensitivity	It mainly reflects the subjects' inferiority complex

**Table 2:** Comparison of the results of the SAS anxiety self-rating scale between the experimental group and the control group before and after the intervention.

	Test group	Control group
*t*	3.734	0.121
Number of people	50	50
Front side	58.45	53.11
Posttest	49.81	53.08

RETRACTED

**Table 3:** Comparison of the results of the SDS self-rating depression scale between the experimental group and the control group before and after the intervention.

	Test group	Control group
*t*	4.22	3.06
Number of people	50	50
Front side	55.02	57.92
Posttest	48.27	53.06

## Data Availability

The data used to support the findings of this study are included within the article.
